# Overall Survival in Patients With Resected Glioblastoma Treated With Adjuvant Therapy: A Retrospective Study in a Public Hospital in Chile

**DOI:** 10.7759/cureus.15105

**Published:** 2021-05-18

**Authors:** Evelyn San Martin, Felipe Carvajal, Alexander Cifuentes, Dandaro Dalmazzo, Freddy Alarcon, Ariel Fariña, Loreto Yañez

**Affiliations:** 1 Radiation Oncology, Servicio de Radioterapia, Hospital Clínico de Magallanes, Punta Arenas, CHL; 2 Radiation Oncology, Servicio de Radioterapia, Instituto Nacional del Cáncer. Universidad de Chile. Santiago, Chile, Santiago, CHL; 3 Radiation Oncology, Servicio de Radioterapia, Instituto Nacional del Cáncer, Santiago, CHL; 4 Radiation Oncology, Servicio de Radioterapia, Instituto Nacional del Cáncer. Universidad Diego Portales, Santiago, CHL; 5 Radiation Oncology, Servicio de Radioterapia, Instituto Nacional del Cancer, Santiago, CHL; 6 Radiation Oncology, Servicio de Radioterapia, Fundación Arturo López Pérez, Santiago, CHL; 7 Radiotherapy, Servicio de Radioterapia, Fundación Arturo López Pérez, Santiago, CHL

**Keywords:** glioblastoma, radiotherapy, temozolomide, adjuvant treatment, survival, chile

## Abstract

Glioblastoma (GB) is the most frequent and aggressive primary tumor of the central nervous system (CNS) in adults. Standard treatment is complete tumor resection followed by concomitant radiochemotherapy (RCT) and subsequent adjuvant temozolomide (TMZ). Information about brain tumors statistics in Latin American countries is scarce, so we aimed to measure the overall survival (OS) of patients with resected GB in a single institution in Chile.

This is a retrospective report of 67 patients treated between 2012 and 2019 with resected GB and who received adjuvant treatment with radiotherapy (RT) with and without TMZ during 2012-2019 in this center (Chilean NCI). Most of them were men (72%), ages > 50 years old (57%), with Karnofsky performance status (KPS) scale ≥ 70% (94%) and recursive partitioning analysis-IV (RPA-IV) (60%). Some 54% received concomitant TMZ and RT. Median OS was 11.4 months, with 1-, 2-, and 5-year OS of 48%,15%, and 3% respectively.

In conclusion, in patients with GB treated with RCT at the NCI, OS was the same as expected from international articles.

Adjuvant RCT therefore is considered the standard of care at NCI.

## Introduction

Glioblastoma (GB) is the most frequent and aggressive primary tumor of the central nervous system (CNS) in adults [1]. Its average age of diagnosis is 64 years old and men have a higher incidence [1-2]. Brain MRI is the preferred imaging study in suspected cases [3]. Histologic diagnosis confirms the GB diagnosis [4], so surgical management has a diagnostic and therapeutic role, with possible neurologic symptom, outcome, and quality of life improvement [5-8].

Standard treatment is complete tumor resection if possible, confirmed with early 24-72 hours after surgery imaging with an MRI with gadolinium [9], followed by concomitant radiochemotherapy (RCT) and subsequent chemotherapy (CT) with temozolomide (TMZ) [10-11]. With this treatment, the median survival is 14.6-21.1 months [11-13]. In addition, poor prognostic factors have been identified, including age, functional status, and the extent of resection, among others [14-15].

In Chile, approximately 80% of the population has public health insurance (FONASA) [16] and this does not ensure TMZ access, mMGMT or other molecular markers in GB. The complete TMZ treatment in Chile exceeds 14,000 dollars [17], so it is a significant barrier for candidates for this therapy, and as a consequence they receive exclusive radiotherapy (RT).

In Chile, this issue has not been published so far and there are scant reports in Latin America [18]. The main objective of this study is to determine the overall survival (OS) of patients with resected GB who received adjuvant therapy with RT (with or without TMZ) at the main Chilean tertiary level of care Oncologic Public Hospital (Chilean NCI) during years 2012-2019.

## Materials and methods

A retrospective cohort study was performed in patients with resected GB and who received adjuvant treatment with RT at the National Cancer Institute (NCI) between 2012 and 2019. The inclusion criteria were: patients with resected GB with histological confirmation based on the CNS WHO tumor classification, aged 18 years of age or more at diagnosis, ECOG Performance status ≤2 at the time of RT planning. Patients with another concomitant malignant neoplasia, who had received systemic treatment for another tumor, who did not complete planned adjuvant RT, who received RT with other than conventional (1.8-2 Gy / fraction) fractionation or those who were treated with palliative intention were excluded.

Data of these patients were obtained from the statistical record service of the NCI. Date of death was acquired from the death records of the Chilean Civil registration. Analyzed variables were: age and sex, performance status (PS) at the beginning of treatment according to the Karnofsky performance status (KPS) scale, recursive partitioning analysis (RPA), date of tumor resection, definitive surgery, the extent of resection, date of initiation of adjuvant treatment with RT, type of adjuvant treatment received (with or without concomitant and/or adjuvant TMD, dose of TMD), and death date or last clinical control. OS was defined as time between start of RT and death. Methylation of the MGMT gene promoter (MGMT) methylation and isocitrate dehydrogenase (IDH) mutation are not reported and unavailable.

The RT technique consisted of 3D conformational RT with a high energy linear accelerator (6-18 MV). Contouring in the first 34 patients was defined as per The Radiation Therapy Oncology Group (RTOG): clinical target volume 1 (CTV1): tumor bed including the T2 FLAIR MRI sequence edema area + 2 cm margin. CTV2: tumor bed + 2 cm margin based on T1 gadolinium MRI. The following 33 patients were treated with a single CTV including the operative bed + residual tumor and a margin of 2.5-3 cm. For the planning target volume (PTV) a margin of 5 mm was added to the CTV. In the first 34 patients, PTV1 prescribed dose was 46 Gy in 23 fractions and a boost to PTV2 up to 60 Gy in fractions of 2 Gy/day. The remaining patient`s PTV received 60 Gy in 30 fractions. Concomitant CT with TMD was administered according to the Stupp trial [10].

For data presentation, descriptive statistics were performed. The groups were compared using Fisher's test for categorical variables and for quantitative variables according to Student's t-test or Wilcoxon-Mann-Whitney test. Kaplan Meier survival analysis was used, with exploratory comparison using the Log rank method and the Cox proportional hazard regression (HR) model to obtain the ratio of risk in univariate and multivariate analysis, considering an α of 5%. Stata / IC®16 (Stata Corp LLC, College station, TX, USA) for Mac software was used.

We use RPA classes in GB (based on four patient variables: age, Karnofsky score, extent of resection, and neurologic function) within the statistical analysis as prognostic classes.

## Results

A total of 358 files with the diagnosis of CNS tumor were reviewed, identifying 82 patients with a diagnosis of GB. Of these, 15 patients were excluded because they did not meet the inclusion criteria and / or consider exclusion (5 did not receive RT, 2 suspended treatment, 4 had palliative intention, 3 had nonconventional 2 Gy per fraction RT fractionation, and 1 was under 18 years old). Finally, a total of 67 patients were included in the analysis. The basal characteristics are detailed in Table 1.

**Table 1:** Overall survival. TMZ, temozolomide; HR, hazard regression

Overall survival	Median (months)	95% IC (months)
Whole cohort	11.4	9.7–14.6
Without TMZ concomitant	9.7	6.1–10.4
With TMZ concomitant	14.6	11.8–20.7
		HR 0.39, (p < 0.001)

Most patients were men (72%), > 50 years (57%), KPS ≥ 70% (94%), and RPA IV (60%).

Regarding surgery, 45% had macroscopic total resection (GTR) and median time from surgery to the start of RT was 50 days.

Globally 54% had concomitant RT TMZ; these patients received 100% of the prescribed standard concomitant dose, but the number of patients receiving TMZ consolidation adjuvant TMZ after RT TMZ is unknown due to lack of data in our clinical records, as many of them received their adjuvant CT outside our institution. The group with exclusive RT included patients with worse prognosis: RPA IV 77% vs 50% (p <0.03) and GTR 41% vs 67% (p <0.04) compared to the RT TMZ group.

For the entire cohort, with a median follow-up of 10.3 (4-70) months, the median OS was 11.4 months, with an OS at 1, 2, and 5 years of 48%, 15%, and 3%, respectively (Table 2).

**Table 2:** Patients and treatment characteristics. TMZ, temozolomide; KPS, Karnofsky score scale; GTR, gross total resection; STR, subtotal resection; RPA, recursive partitioning analysis; RT, radiotherapy

Variables	Cases	%
Total patients	67	100
Age		
> 50 years old (%)	38	57
< 50 years old (%)	29	43
Years [median (range)]	50 (range 20-76)	
Gender		
Female (%)	19	28
Masculine (%)	48	72
KPS before RT		
≥ 70 (%)	63	94
< 70 (%)	4	6
Extent of resection		
GTR	30	45
STR	37	55
RPA		
III	25	37
IV	40	60
V	2	3
Time from surgery to RT		
Days [median (range)]	50 (range 31-156)	
TMZ concomitant with RT		
Yes	36	54
No	31	46

Differences in OS were identified when patients were stratified according to RT treatment with concomitant TMZ vs without TMZ, presenting a median OS of 14.6 months vs 9.7 months, a 2-year OS of 26% vs 4%, and 5-year OS of 10% vs 2%, respectively (Figure 1). A significant better survival was observed on univariate analysis (Table 2) with concomitant TMD (HR 0.48, p < 0.001), but this lost significance in the multivariate analysis (Table 3).

**Figure 1:** Overall survival of the cohort.

**Table 3:** Multivariate analysis. HR, hazard regression; KPS, Karnofsky performance status; RPA, recursive partitioning analysis; GTR, gross total resection; STR, subtotal resection

Variable	P Univariate	HR	P Multivariate	HR
Age (≥ 50 vs < 50 years old)	0,01	2,1	0,03	3,8
Gender	0,8	1,1		
KPS (< 70 vs ≥ 70)	0,2	1,9		
RPA (≥ IV vs III)	0,02	2	0,6	0,7
Resection (GTR vs STR)	0,01	0,4	0,001	0,3
Concomitant TMZ	0,001	0,4	0,09	0,6
Time from surgery to RT	0,06	0,5		
(≥ 2 vs < 2 months)				

Of the entire sample, 18 patients had RPA 1 and TMZ. In this subgroup, the median OS was 14.6 months with OS at 1, 2, and 5 years of 80%, 39%, and 15%, respectively. Patients with RPA-III, IV, and V had a median survival of 14.1 vs 10.1 vs 7.4 months respectively (p < 0.02) (Figure 2). Considering the other variables, patients with GTR had better survival than STR (p < 0.001) and those <50 years better than ≥50 years (p < 0.009). The rest of the variables did not show significant differences.

After multivariate analysis, the extent of resection and the age of the patient remained significant, while for concomitance there was only a trend (HR 0.6 95% CI 0.33-1.09).

## Discussion

This is the first published analysis with Chilean data of survival in GB patients. Ours results are consistent with international experiences.

Several studies have been carried out to obtain better oncological results in this pathology. The pivotal study, which defines the current standard of treatment, is a randomized Phase III clinical trial conducted by the EORTC Group [10], in which RT alone was compared to concomitant TMZ for seven weeks followed by adjuvant for six cycles. Some 573 GBM patients were included in which 82% underwent surgery, 85% completed the concomitant scheme, but only 47% completed the adjuvant cycles. The RCT has a HR of death of 0.63 (95% CI 0.52-0.75, p = 0.001) vs RT alone. The two-year survival was 27.2% (95% CI 22.2%-32.5%) with combined therapy vs 10.9% (95% CI 7.6%-14.8%) with RT alone. At five years, the OS is 9.8% vs 1.9%, respectively. Progression-free survival (PFS) was 6.9 months (95% CI 5.8-8.2) vs 5 months (95% CI 4.2-5.5). Among the adverse effects, severe myelosuppression occurred in 16% of patients, but only 5% discontinued therapy [10-11].

A Cochrane systematic review demonstrated that the use of TMZ concomitant to RT vs RT alone in patients with high-grade gliomas was associated with better OS (HR 0.60, 95% CI 0.46-0.79, p = 0.0003) and better PFS (HR: 0.63, 95% CI 0.43-0.92, p = 0.02). The benefit was greater for the concomitant and adjuvant therapy regimens, without demonstrating benefit in the concomitant regimen without adjuvant treatment. The risk of infections, fatigue, and hematological complications was higher with TMZ [19].

We can observe that the two-year and five-year OS in patients who received concomitant TMZ in our cohort is similar to that published by Stupp et al. [10]. However, the median OS in the group with exclusive RT was lower than the control group of that study, which can be explained by selection bias, since group with exclusive RT in our cohort included patients with worse prognostic factors. Univariate analysis showed higher survival in patients with concomitant RT TMZ, but significance was lost in multivariate analysis, probably accounting for bias.

Regarding the extent of tumor resection, we observed that those who were treated with GTR had a 70% survival benefit compared to those with STR. These results are consistent with what has been published internationally. A recent meta-analysis showed a 35% lower risk of mortality in patients treated with GTR vs STR [20]. This could be related to the significant delay in the start of adjuvant treatment that we observed, with a median of close to two months between surgery and RT. In this context, the absence of tumor residue during this interval could be important. A study based on the NCDB data showed that even in patients with GTR, OS decreases if RT is started with a delay greater than eight weeks (HR 1.23, p = 0.007), therefore reducing this interval to 4-8 weeks could be considered optimal [21]. Finally, we observed better survival in patients under 50 years of age, similar to previously published articles [22].

Chilean public system has economic limitations so glioblastoma tumor patients do not have full diagnostic characterization with molecular markers, or access to TMZ, so response to therapy and prognosis in our series is not accurately described as in other publications [23-24]. It would have been interesting to report toxicity, but this information was not readily and reliably available.

Although the design of our study does not allow conclusions other than consistent results with previously published international phase III trials, it has the value of reporting the results of a single institution with limited access to TMZ.

## Conclusions

Despite the limitations faced by resected GB patients in our public health system, those who received RT with concomitant TMZ, OS is representative of the phase III Stupp trial. It is important to achieve a GTR, optimize the interval from surgery to initiation of RT TMZ adjuvant therapy, and there is a need to emphasize an improved access to TMZ for patients with public health insurance.

## References

[1] Ostrom QT, Gittleman H, Truitt G, Boscia A, Kruchko C, Barnholtz-Sloan JS (2018). CBTRUS statistical report: primary brain and other central nervous system tumors diagnosed in the United States in 2011-2015. Neuro Oncol.

[2] Thakkar JP, Dolecek TA, Horbinski C, Ostrom QT, Lightner DD, Barnholtz-Sloan JS, Villano JL (2014). Epidemiologic and molecular prognostic review of glioblastoma. Cancer Epidemiol Biomarkers Prev.

[3] (2005). Diagnostic imaging: brain. Am J Neuroradiol.

[4] Reifenberger G, Collins VP (2004). Pathology and molecular genetics of astrocytic gliomas. J Mol Med (Berl).

[5] Hentschel SJ, Lang FF (2003). Current surgical management of glioblastoma. Cancer J.

[6] Ammirati M, Vick N, Liao YL, Ciric I, Mikhael M (1987). Effect of the extent of surgical resection on survival and quality of life in patients with supratentorial glioblastomas and anaplastic astrocytomas. Neurosurgery.

[7] Sawaya R, Hammoud M, Schoppa D, Hess KR, Wu SZ, Shi WM, Wildrick DM (1998). Neurosurgical outcomes in a modern series of 400 craniotomies for treatment of parenchymal tumors. Neurosurgery.

[8] Brown PD, Maurer MJ, Rummans TA (2005). A prospective study of quality of life in adults with newly diagnosed high-grade gliomas: the impact of the extent of resection on quality of life and survival. Neurosurgery.

[9] Weller M, Le Rhun E, Preusser M, Tonn JC, Roth P (2019). How we treat glioblastoma. ESMO Open.

[10] Stupp R, Mason WP, van den Bent MJ (2005). Radiotherapy plus concomitant and adjuvant temozolomide for glioblastoma. N Engl J Med.

[11] Stupp R, Hegi ME, Mason WP (2009). Effects of radiotherapy with concomitant and adjuvant temozolomide versus radiotherapy alone on survival in glioblastoma in a randomised phase III study: 5-year analysis of the EORTC-NCIC trial. Lancet Oncol.

[12] Lai A, Tran A, Nghiemphu PL (2011). Phase II study of bevacizumab plus temozolomide during and after radiation therapy for patients with newly diagnosed glioblastoma multiforme. J Clin Oncol.

[13] Roh TH, Park HH, Kang SG (2017). Long-term outcomes of concomitant chemoradiotherapy with temozolomide for newly diagnosed glioblastoma patients: a single-center analysis. Medicine (Baltimore).

[14] Wang TJ, Jani A, Estrada JP (2016). Timing of adjuvant radiotherapy in glioblastoma patients: a single-institution experience with more than 400 patients. Neurosurgery.

[15] Lacroix M, Abi-Said D, Fourney DR (2001). A multivariate analysis of 416 patients with glioblastoma multiforme: prognosis, extent of resection, and survival. J Neurosurg.

[16] (2020). Fonasa [Internet]. https://www.fonasa.cl/sites/fonasa/conoce-fonasa.

[17] Lista de Precios 2019 Lista de Precios 2019. MSD Latinoamérica [Internet]. http://www.msdlatinamerica.com/chile/listadeprecios.pdf.

[18] Piñeiro N, Perna A, Baldizzoni M (2014). Estudio de una cohorte uruguaya de portadores de glioblastoma tratados con radioterapia y temozolamida. Arch Med Intern.

[19] Hart MG, Grant R, Garside R, Rogers G, Somerville M, Stein K (2013). Temozolomide for high grade glioma. Cochr Datab Syst Rev.

[20] Jackson C, Choi J, Khalafallah AM (2020). A systematic review and meta-analysis of supratotal versus gross total resection for glioblastoma. J Neurooncol.

[21] Buszek SM, Al Feghali KA, Elhalawani H (2020). Optimal timing of radiotherapy following gross total or subtotal resection of glioblastoma: a real-world assessment using the National Cancer Database. Sci Rep.

[22] Azab A, Alsayegh N, Kashkari O (2020). Factors affecting survival in glioblastoma: a 10-year single-center experience from Saudi Arabia. Gulf J Oncol.

[23] Zreik J, Moinuddin FM, Yolcu YU, Alvi MA, Chaichana KL, Quinones-Hinojosa A, Bydon M (2020). Improved 3-year survival rates for glioblastoma multiforme are associated with trends in treatment: analysis of the national cancer database from 2004 to 2013. J Neurooncol.

[24] Strowd RE (2020). In the midst of crisis, a great opportunity. Neuro Oncol.

